# A Transformer-Based Network for Change Detection in Remote Sensing Using Multiscale Difference-Enhancement

**DOI:** 10.1155/2022/2189176

**Published:** 2022-08-13

**Authors:** Gulinazi Ailimujiang, Yiliyaer Jiaermuhamaiti, Huxidan Jumahong, Huiling Wang, Shuangling Zhu, Pazilaiti Nurmamaiti

**Affiliations:** ^1^College of Network Security and Information Technology, YiLi Normal University, Yining 835000, China; ^2^College of Electronics and Engineering, YiLi Normal University, Yining 835000, China

## Abstract

Recently, transformer-based change detection methods have achieved remarkable performance by sophisticated architectures for extracting powerful feature representations. However, due to the existence of various noises in bitemporal images, there are problems such as loss of semantic objects and incompleteness that will occur in change detection. The existing transformer-based approaches do not fully address this issue. In this paper, we propose a transformer-based multiscale difference-enhancement U-shaped network and call it TUNetCD, for change detection in remote sensing. The encoder, which is composed of a multilayer Swin-Transformer block structure, can extract multilevel feature maps, further enhance these multilevel feature maps using a Swin-Transformer feature difference map processing module, and finally obtain the final change map using a lightweight decoder. We conducted comprehensive experiments on two publicly available benchmark datasets, LEVIR-CD and DSIFN-CD, to verify the effectiveness of the method, and our method outperformed other advanced transformer-based methods.

## 1. Introduction

The goal of remote sensing image change detection (CD) is to generate a binary change map (BCM) by comparing and analyzing two images taken at different times of day for the same area. Each pixel in the binary change map image consists of a 0 or a 1, corresponding to a change or no change in that pixel's position. The definition of change detection varies depending on the task. It is used for tasks such as urban area change detection [1, 2], environmental detection [3, 4], land use detection [5, 6], and disaster assessment [7]. Change detection methods that have been continuously updated in recent years are widely used in a variety of fields and are attracting the attention of more scholars.

Convolutional neural networks (CNNs) have gained wider applications in several fields of computer vision in recent years, such as image classification [5, 6], target detection [7], semantic segmentation [8], and face recognition [9]. CNN-based CD algorithms have also made significant strides [8, 10–19]. Zhan et al. used a Siamese convolutional network in the CD task to extract two feature maps of diachronic images by two parallel weight-sharing convolutional branches and then compared the feature thresholds. Following that, many CD methods adopted this architecture [10]. Rahman F et al. proposed the Siamese network approach, which eliminates the threshold comparison with a decision network [11]. Following the success of fully convolutional networks (FCN) [8] and U-net [12] in image segmentation, its various variants now provide an effective method for change detection. Daudt et al. were the first to use FCN for CD tasks, proposing three FCN frameworks: FC-EF, FC-Siam-Conc, and FC-Siam-Diff [13]. However, because CNNs are more focused on local information, the extraction of global features is weak. Scholars have proposed a series of approaches to this problem. To extract multiscale features, Chen et al. proposed using ResNet as the encoder backbone and adding a pyramid self-attention structure [14]. Chen et al. then utilized the dual attention module to obtain long-range results [15]. Peng et al. proposed UNet++, which learns multiscale feature maps using dense skip connections and controls gradient convergence with residual blocks [16]. FCN was used by Zhang et al. to extract deep features, which were then fed into the proposed deep-supervised image fusion network (DSIFN) [17]. To improve encoder and decoder performance, Fang et al. proposed a densely connected U-type Siamese network [18].

The transformer proposed by Vaswani et al. was first used with great success on the neural machine translation (NMT) task of natural language processing (NLP) [19]. It was then widely used in various NLP fields. Dosovitskiy et al. proposed the vision transformer (ViT) as the first pure transformer algorithm, which was first used for computer vision (CV) tasks and proved to be effective in image classification tasks [20]. Meanwhile, due to transformer's superior semantic representation capability over CNN, many scholars applied the ViT method to various CV tasks and achieved comparable or better results than CNN. The Swin-Transformer shifted windowing scheme proposed by Liu et al. divides the window into multiple local windows and computes the self-attention hierarchy transformer within the local window [21]. This method effectively reduces the computational complexity of self-attention while also increasing accuracy. Xie et al. proposed combining the ViT encoder with a lightweight multilayer perceptron (MLP) decoder to form SegFormer, an efficient semantic segmentation framework that obtains multiscale features while avoiding complex decoders [22]. Bandara and Patel proposed unifying a hierarchically structured ViT encoder and an MLP decoder of the Siamese network framework to obtain multiscale long-range features [23]. The success of ViT and Swin-Transformer on various CV tasks, including CD, has aided in the development of further CD capabilities.

We designed a new network named transformer-based multiscale difference-enhancement U-shaped networks after being inspired by the previous work (TUNetCD).

Firstly, coregistered image pairs are concatenated as an input for the improved TUNetCD network, which can generate information using both global and fine-grained information. Second, numerous studies have demonstrated that shallow layers on the encoder side output fine-grained features, whereas deep layers output coarse-grained features. TUNetCD is being used to learn multiscale and semantic levels of visual feature representations to fine-tune the spatial details. To solve the CD task, we adopted a pure Swin-Transformer network with a U-shaped structure. Because TUNetCD's basic unit is a Swin-Transformer block, it can obtain both local fine-grained features.

The following are the main contributions of this paper:

1. To build the encoder and feature difference map processing module, we proposed TUNetCD, a hierarchical U-shaped image change detection framework with LeWinTransformer as the main module.
2. To capture the local and global correlations of hierarchical multilevel features, we proposed a feature difference map processing module based on the LeWinTransformer block.
3. The superior experimental results on change detection datasets demonstrate the effectiveness and robustness of the proposed TUNetCD.

## 2. Related Work

In this section, the CNN framework for CD, the transformer mechanism, and the FCN method based on consistency regularization will be briefly illustrated.

### 2.1. CNN-Based CD Methods

In recent years, deep learning (DL) algorithms have attracted much attention. Deep learning models can learn multiple levels of representation and abstraction to help understand images and extract semantic information from them. In the field of remote sensing images processing, deep learning has also shown excellent performance [24] and is widely used in problems such as the remote sensing image change detection problem [25].

Most of the DL networks for CD tasks are based on convolutional neural networks. CNN-based CD methods usually enhance the semantic representation ability of network by changing the network structure, optimizing loss function, adding attention mechanism, and so on.

In terms of network structure, Zhan et al. [10] used a Siamese convolutional network in the CD task to extract two feature maps of diachronic images by two parallel weight-sharing convolutional branches and then compared the feature thresholds. Following that, many CD methods adopted this architecture. Daudt et al. [13] designed the first end-to-end training CD method and proposed three effective FCNN-based architectures. In [13], FC-EF concatenates the bitemporal images as the input of the network, while FC-Siam-conc and FC-Siam-diff leverage a Siamese structure, which can directly process bitemporal images. The most intuitive way to reduce the inherent locality of convolution operation is to increase the reception field. To extract multiscale features, Chen and Shi [14] proposed spatial–temporal attention neural network (STANet), using residual nets (ResNet) as the encoder backbone and adding a pyramid self-attention structure. Chen et al. [15] proposed dual attentive fully convolutional Siamese networks (DASNet) and then utilized the dual attention module to obtain long-range results. Compared with the shallow networks, STANet and DASNet have stronger feature extraction capability. Huang et al. [6] proposed dense connections (DenseNets) are built from dense blocks and pooling operations, where each dense block is an iterative concatenation of previous feature maps. Among them, the UNet based on fully convolutional networks is the most popular and has become one of the standard CNN architectures for CD tasks with many extensions [24]. By adding a skip connection between encoder and decoder, UNet can better integrate deep semantic information and shallow spatial information, improving the accuracy of CD. Fang et al. [18] proposed the combination of Siamese network and UNet++ (SNUNet-CD) added dense connections between the features of different layers, so as to enhance the capability of the CD network.

In the remote sensing images, the changed pixels are far less than the unchanged pixels, so there exists a serious data imbalance in the CD task. Many scholars solved this problem by optimizing the loss function so that the changed and unchanged pixels participate in the loss calculation in the same proportion. Zhan et al. [10] proposed a weighted contrastive loss function, which increased the weight of the changed pixels in the loss calculation. STANet [14] and DASNet [15] further optimized the weighted contrastive loss function, and they proposed batch-balanced contrastive loss function and weighted double-margin contrastive loss function. In SNUNet proposed by Fang et al. [18], a hybrid loss function was used to optimize the network.

Since attention mechanism has achieved remarkable results in the CV task, many scholars have introduced attention mechanism into CD task. Chen et al. [15] introduced a dual attention module into the CD task to learn features that contain both channel information and spatial information. Fang et al. [18] proposed an ensemble channel attention module (CAM) to fuse the features of various levels, so as to generate stronger change features. In order to detect changes with different sizes, Chen and Shi [14] proposed a pyramid spatial–temporal attention module, which can extract features from different scales. Peng et al. [26] designed a dense attention method to extract richer and more effective features. Chen et al. [27] introduced the transformer into the field of CD for the first time and proposed bitemporal image transformer (BiT). First of all, BiT uses CNN to generate semantic features. Second, BiT leverages a transformer module to further process CNN features. Finally, BiT uses a prediction head module to generate the change maps.

Although the above methods have improved the ability of CD network to a certain extent, due to the inherent locality of convolution operation, the CNN-based methods cannot effectively extract long-term global features, thus limiting the ability of CD network. Unlike the previous methods, this article attempts to explore the potential of pure transformer network for the CD task.

### 2.2. Transformer-Based CD Methods

Dosovitskiy et al. [20] proposed the ViT as the first pure transformer algorithm. In image classification, ViT achieves comparable results with CNN-based algorithms. However, one drawback of ViT is that we need to pretrain ViT on a larger dataset, which makes the training of ViT inconvenient. The computational complexity of ViT is quadratic to the size of the input image, so ViT is not suitable for the dense vision tasks. Liu et al. [21] proposed that Swin-Transformer used shifted windowing scheme to calculate self-attention in a local window, which not only reduced the computational complexity but also acquired the best results in several CV tasks. Motivated by ViT, BiT [27] firstly proposed a bitemporal image transformer network for effectively modeling spatial–temporal contexts, which innovatively proved the enhancing ability by combining a CNN and a transformer. A transformer-based Siamese network architecture (abbreviated by ChangeFormer) [23] is a hierarchical transformer in a Siamese network with a lightweight decoder, and it shows that good results can still be obtained without relying on the convolution operation. However, these mentioned transformer-based CD frameworks are merely capable of capturing global interdependencies of single-scale objects within each transformer layer, which tend to lose robustness in rich spatial scenes of remote sensing images. The local context information is essential for image change detection tasks since the neighborhood of a change pixel can be leveraged to restore its information, but previous works suggest that transformer shows a limitation in capturing local dependencies.

Inspired by the success of LeWin transformer in dense vision tasks, we introduce the LeWin transformer into the CD task and propose TUNetCD that is a pure LeWin transformer network with a multiscale difference-enhancement U-shaped structure. In our proposed method, we not only retain the original feature maps but also adopt the feature difference maps to model multiscale and multidepth change information, which will enhance the change intensity.

## 3. Methods

### 3.1. Framework Overview

As shown in Figure 1, the proposed NET consists of three major components: a hierarchical transformer encoder in a U-shape network to extract multiscale features, a feature difference map processing module, and a decoder. The LeWinTransformer block serves as the foundation for the first two components. Through the overlapped image patches, the encoder extracts hierarchical features. *T*, the feature difference map processing module, is used to improve the information of the changed areas. To predict the change map, the decoder aggregates the multilevel feature difference maps.

{*X*_1_, *X*_2_} ∈ *R*^*H*×*W*×3^ are the input bitemporal feature maps, where *H*, *WW*, and *C* are height, width, and channel dimension of the feature map *X*_1_*X*_2_. We'll get the input feature map *X* ∈ *R*^*H*×*W*×6^ feature map after concatenating *X*_1_ and *X*_2_. After entering it into the encoder *X*, we will first enter to the Overlap Patch Embedding module to convert *X* into image tokens and then use hierarchical LeWinTransformer to generate multilevel features *F*_enc_^*i*^ ∈ *R*^(*H*/2^*i*+1^)×(*W*/2^*i*+1^)×*C*^*i*^^, where *i*={1,2,3,4} and *C*^*i*+1^ > *C*^*i*^, which will be further processed through the feature difference map processing module to generate multilevel features *F*_diff_^*i*^ ∈ *R*^(*H*/4)×(*W*/4)×*C*_emb_^. The features are then passed to the decoder, which predicts the binary change map *F*_*cm*_ ∈ *R*^*H*×*W*×2^.

### 3.2. Hierarchical Transformer Encoder

#### 3.2.1. Overlapped Patch Merging

We used overlapping patch merging to tokenize the feature map and implemented downsampling to reduce computational consumption. In the Overlapped Patch Merging module, if given a hierarchical feature map *F*^*i*^ ∈ *R*^(*H*/2^*i*+1^)×(*W*/2^*i*+1^)×*C*^*i*^^ (*i* denotes the *i*_*th*_ stage), it unifies patch into feature map size as F^*i*+1^ ∈ *R*^(*H*/2^*i*+1^)×(*W*/2^*i*+1^)×*C*^*i*+1^^ and then iterates for any other features map in the hierarchy. As a result, we defined *K* as the patch size, *S* is the stride between two adjacent patches, and *P* is the padding size. We utilized a conv2D layer with *K*=7, *S*=4, and *P*=3 for the initial merging, and *K*=3, *S*=2, and *P*=1 for the rest.

#### 3.2.2. LeWinTransformer Block

ViT is confronted with two major challenges: (1) when calculating global attention, self-attention must pay attention to all tokens, and the calculation cost increases quadratically with the number of tokens; (2) local context information is critical for all types of CV tasks, and the neighborhood of a change pixel must have significant differences. ViT has a limitation when it comes to capturing local dependencies.

Swin-Transformer is a module that replaces standard multihead self-attention based on (shifted) window multihead self-attention ((S) W-MSA). Other layers remained unchanged. We use the LeWinTransformer module, which is based on (S) W-MSA.

The locally enhanced window (LeWin) transformer block, as shown in the upper left of Figure 1, can obtain long-range dependencies by using the self-attention mechanism in transformer or by adding the LeFF (locally enhanced feedforward network) module of the conversion operator to obtain local context information. Specifically, (*l* − 1)*th* assumes that, in the output feature *F*^*l*−1^ of the LeWinTransformer block, our LeWinTransformer block consists of two main parts: (1) nonoverlapping window multihead self-attention (W-MSA) and (2) locally enhanced feedforward network (LeFF). The calculation formulas of the block are as follows:

(1) $$\begin{array}{c} {\hat{F}}^{l}=W-MSA\left(LN\left(F^{l-1}\right)\right)+F^{l-1},\\ F^{l}=LeFF\left(LN\left({\hat{F}}^{l}\right)\right)+{\hat{F}}^{l}, \end{array}$$

where ${\hat{F}}^{l}$ and *F*^*l*^ are the outputs of the W-MSA module and LeFF module, respectively. LN represents the layer normalization.

The feature maps are partitioned into nonoverlapping windows, and each patch is calculated within each window.

*(1) Window Multihead Self-Attention (W-MSA) Module*. The W-MSA module divides the feature map into several nonoverlapping windows, and each window size is *N* × *N*. The feature patches then calculated self-attention within each window. As shown in Figure 2, given the input feature map *F*_in_ ∈ *R*^*H*×*W*×*C*^, where *H*, *W*, and *C* are height, width, and channel dimension of the feature map, *F*_in_ are partitioned into *N* × *N* nonoverlapping windows. Therefore, we define *F*_in_^*i*^ ∈ *R*^*N*×*N*×*C*^ as the feature of the *i*_*th*_ window, where *i* ∈ {1,2,…, *Z*} and *Z*=(*H·W*/*N*^2^)*F*_in_^*i*^ are flattened and transposed into *F*^*i*^ ∈ *R*^*N*^2^×*C*^. Subsequently, we perform self-attention on *F*^*i*^ in each window. Firstly, *F*^*i*^ is linearly projected into query *Q*^*i*^ ∈ *R*^*N*^2^×*C*^, key *K*^*i*^ ∈ *R*^*N*^2^×*C*^, and value *V*^*i*^ ∈ ℝ^*N*^2^×*C*^ matrices.

(2) $$\begin{array}{c} Q^{i}=F^{i}\cdot W^{Q}\\ K^{i}=F^{i}\cdot W^{K},\\ V^{i}=F^{i}\cdot W^{V}, \end{array}$$

where *W*^*Q*^, *W*^*K*^, and *W*^*V*^ are learnable parameters and have the same dimensions of *R*^*C*×*C*^*R*^*C*×*C*^, representing the weights of three linear projection layers, respectively. Second, we split *Q*^*i*^, *K*^*i*^, and *V*^*i*^ into *h* heads along the channel dimension, respectively. Then, they can be expressed as *Q*^*i*^=[*Q*_1_^*i*^, *Q*_2_^*i*^,…, *Q*_*h*_^*i*^], *K*^*i*^=[*K*_1_^*i*^, *K*_2_^*i*^,…, *K*_*h*_^*i*^], and *V*^*i*^=[*V*_1_^*i*^, *V*_2_^*i*^,…, *V*_*h*_^*i*^]; the head dimension is *d*_*h*_=(*C*/*h*). The computation of *k*_*th*_ head self-attention in nonoverlapping windows can then be formulated as follows:

(3) $$\begin{array}{c} \text{Self}-\text{Attention}\left(Q_{k}^{i},K_{k}^{i},V_{k}^{i}\right)=\text{softmax}\left(\frac{Q_{k}^{i}\cdot K_{k}^{i}}{\sqrt{d_{h}}}\right)V_{k}^{i}, \end{array}$$

where *Q*_*k*_^*i*^, *K*_*k*_^*i*^, and *V*_*k*_^*i*^ represent the projection matrices of the query, key, and value for the *k*_*th*_ head, respectively. Third, the output tokens *F*_out_^*i*^ ∈ *R*^*N*^2^×*C*^ of the *i*_*th*_ window can be obtained by

(4) $$\begin{array}{c} F_{\text{out}}^{i}=\overset{h}{\underset{k=1}{\text{Concat}}}\left(\text{Self}-\text{Attention}\left(Q_{k}^{i},K_{k}^{i},V_{k}^{i}\right)\right)W^{\text{out}}+P, \end{array}$$

where Concat(*·*) denotes the concatenating operation and *P* ∈ *R*^*N*^2^×*C*^ is the relative position bias. They are taken from $\hat{P}\in R^{\left(2N-1\right)\times \left(2N-1\right)}$ with learnable parameters, and *W*^out^ ∈ *R*^*C*×*C*^ are learnable parameters. Then, we reshape *F*_out_^*i*^ to obtain the output window feature map *F*_*o*_^*i*^ ∈ *R*^*N*×*N*×*C*^. Finally, we merge all the patch representations {*F*_*o*_^1^, *F*_*o*_^2^, *F*_*o*_^3^,…, *F*_*o*_^*Z*^} to obtain the output feature maps *F*_out_ ∈ *R*^*H*×*W*×*C*^.

*(2) Feedforward Network (FFN)*. As illustrated in Figure 3, Swin-Transformer's feedforward network (FFN) is composed of a 1 × 1 conv layer with a GELU activation, a depth-wise 3 × 3 conv layer with a GELU activation, and another 1 × 1 conv layer.

*(3) Locally Enhanced Feedforward Network (LeFF)*. The standard ViT's FFN has limited ability to leverage local context. To address this issue, we employed LeFFN to improve local context information. As shown in Figure 1, we first applied a linear projection layer to each token to increase the dimension of its features. The tokens were then reshaped into 2D feature maps, and local information was captured using a depth-wise convolution. The features were then flattened back to tokens, and the channels were shrunk via another linear layer to match the dimension of the input channels. After each linear/convolution layer, we used GELU as the activation function.

### 3.3. Feature Difference Map Processing Module

We obtained four multiscale feature maps from the encoder in the feature difference map processing module. The features with the smallest scale are considered high-level features because they contain rich semantic and attribute information. The sizes of the other three features gradually transition from high-level features to low-level features from small to large, and the features of which they primarily consist also change to texture and detailed information of ground objects. We can use feature difference map processing to take advantage of the interaction between high-level features and low-level features, guide the categories and attributes of low-level features with high-level features, and provide detailed information for high-level features. We used LeWinTransformer in the feature difference map processing module to strengthen and suppress information in each feature. In contrast to convolutions, the LeWinTransformer can capture long-range dependencies and attend to diverse information from a global perspective.

#### 3.3.1. MLP

We first processed each multiscale feature through an MLP layer to unify the channel dimension to value *C*_*eb*  *d*_.

(5) $$\begin{array}{c} {\hat{F}}_{\text{out}}^{i}=\text{Linear}\left(C_{i},C_{eb\;d}\right)\left(F_{\text{out}}^{i}\right)\forall i, \end{array}$$

where *C*_*eb*  *d*_ denotes the embedding dimension.

#### 3.3.2. LeWinTransformer

(6) $$\begin{array}{c} F_{l\_\text{diff}}^{i}=\text{LeWinTransformer}\left({\hat{F}}_{\text{out}}^{i}\right)\forall i. \end{array}$$

#### 3.3.3. Upsampling

We finally unsampled each multiscale feature to size of (*H*/4) × (*W*/4) as follows:

(7) $$\begin{array}{c} \left(F_{l\_\text{diff}}^{i}\right)\forall iF_{\text{diff}}^{i}=\text{Upsample}\left(\left(\frac{H}{4},\frac{W}{4}\right),{}^{\prime \prime }\text{bilinear}{}^{\prime \prime }\right)\left(F_{l\_\text{diff}}^{i}\right)\forall i. \end{array}$$

### 3.4. Decoder

#### 3.4.1. Concatenation and Fusion

These feature maps with uniform channel dimension sizes are concatenated and then fused via an MLP layer as follows:

(8) $$\begin{array}{c} F_{C}=\text{Linear}\left(4C_{ebd},C_{ebd}\right)\left(\text{Cat}\left(F_{\text{diff}}^{1},F_{\text{diff}}^{2},F_{\text{diff}}^{3},F_{\text{diff}}^{4}\right)\right). \end{array}$$

#### 3.4.2. Upsampling and Classification

We upsampled the fused feature map *F*_*c*_ to the size of *H* × *W* by utilizing a transposed conv2d layer with stride of 4 and kernel size of 3. Finally, the upsampled feature map was processed through a MLP layer to predict the change mask *CM*=ℝ^*H*×*W*×2^. This process can be formulated as follows:

(9) $$\begin{array}{c} F=\text{ConvTranspose}2\;D\left(S=4,K=3\right)\left(F_{C}\right), \end{array}$$

(10) $$\begin{array}{c} CM=\text{Linear}\left(C_{eb\;d},2\right)\left(F\right). \end{array}$$

## 4. Experimental Setup

### 4.1. Datasets

For our experts, we used two publicly available CD datasets: LEVIR-CD [14] and DSIFN-CD [17]. The LEVIR-CD dataset is a building CD dataset with RS image pairs of resolution. We use 2048 patches as test datasets, 1024 patches as val datasets, and 7120 patches as train datasets, and we cropped nonoverlapping patches of size. The DSIFN dataset is a general CD dataset that includes changes to various landcover objects. We divided the original train dataset, val dataset, and test dataset into nonoverlapping patches of 14400, 1360, and 192 patches in the three sets of train dataset, val dataset, and test dataset, respectively.

### 4.2. Implementation Details

We implemented our model in Pytorch using NVIDIA 3070 GPU. We randomly initialized the network during training and applied data augmentation through random flip, random rescale (0.8–1.2), and random crop. We trained the models using the Cross-Entropy (CE) Loss and AdamW optimizer with weight decay equal to 0.01 and beat values equal to (0.9, 0.999). The learning rate is initially set to 0.0001 and linearly decays to 0 util trained for 200 epochs. We used a batch size of 2 to train the model.

### 4.3. Performance Metrics

To compare the performance of our model with SOTA methods, we reported F1 and Intersection over Union (IoU) scores with regard to the TUNetCD as the primary quantitative indices. Additionally, we reported precision and recall of the change category.

In order to quantitatively evaluate the performance of our proposed method, precision (P), recall (R), F1-score, and Intersection over Union (IoU) are utilized to compare the labels and our results, which are calculated as follows:

(11) $$\begin{array}{c} P=\frac{TP}{TP+FP}, \end{array}$$

(12) $$\begin{array}{c} R=\frac{TP}{TP+FN}, \end{array}$$

(13) $$\begin{array}{c} F1=2\times \frac{P\times R}{P+R}, \end{array}$$

(14) $$\begin{array}{c} IoU=\frac{TP}{TP+FP+FN} \end{array}$$

where true positive (TP) and true negative (TN) denote the number of changed and unchanged pixels detected correctly, respectively. False positive (FP) and false negative (FN) denote the number of changed and unchanged pixels detected incorrectly, respectively.

## 5. Results and Discussion

### 5.1. Comparative Experiments

In this section, we analyzed the results of our proposed TUNetCD method with the other four new methods on two CD datasets.

STANet [14] is a Siamese-based spatial–temporal attention network for CD.

SNUNet [17] is a multilevel feature concatenation method, in which a densely connected (NestedUNet) Siamese network is used for change detection.

The transformer-based method (BIT) [27] is used for the first time in the CD task, which obtains feature maps in a Siamese network with a ConvNet structure and then passes through a transformer encoder-decoder network to enhance the semantic tokens with the context-information semantic tokens, and finally the refined features are obtained to predict the change map.

ChangeFormer [23] is a transformer-based Siamese network architecture. It leverages the hierarchically structured transformer encoder and multilayer perception (MLP) decoder in a Siamese network architecture for change detection.

Table 1 presents the results of the aforementioned four methods on the test-sets of LEVIR-CD [14] and DSIFN-CD [17]. As can be seen from the table, the proposed TUNetCD network achieves better CD performance in four terms of precision, recall, F1, and IoU metrics. In particular, our TUNetCD improves previous baseline ChangeFormer in precision/recall/F1/IoU by 1.18/3.18/1.96/3.74 percentage (%) and 0.46/0.18/1.28/0.5 percentage (%), for LEVIR-CD and DSIFN-CD, respectively.

### 5.2. Ablation Study

It is well known that many factors can affect the model results, such as network structure and parameter initialization method. In this section, we mainly research the influences of feature difference map processing block on the TUNetCD model. For the factor, we conducted ablation experiments on the LEVIR-CD and DSIFN-CD datasets.

Impact of feature difference map processing block: the feature difference map processing block contains a LeWinTransformer block. In experiments, we verify the validity of the block.

We gradually added LeWinTransformer block to the baseline. The detailed structure of the baseline is shown in Figure 4. Except for the LeWinTransformer block, everything looks similar to Figure 1 of this paper. We conducted an ablation experiment on two datasets. There are two experiments: baseline, baseline + LeWinTransformer block.  Table 2 shows the results of these two experiments. It can be seen that, without adding the LeWinTransformer block, the network performs poorly, with F1 of 89.53% and 84.98% on the two datasets LEVIR-CD and DSIFN-CD, respectively, which is a huge gap compared to other models that join the LeWinTransformer block.

The addition of the LeWinTransformer block to baseline is our proposed network. With the addition of the LeWinTransformer block module, the semantic information and location information in the feature maps are fully accessible at each level, facilitating the model in detecting the precise change regions. Due to the characteristics of P-R curves, in general, the detection rate tends to be low when the accuracy is high. Compared with the baseline and baseline + LeWinTransformer block, the P metric of the TUNetCD network achieves good results, although the *R* metric decreases slightly. F1 and IoU metrics achieve good performance, which proves that the LeWinTransformer block module proposed by TUNetCD can be used in combination with other modules to make further improvements in network performance.

## 6. Conclusion

The network consists of three parts to explore the potential of a pure transformer-based U-shaped structure: a hierarchical Swin-Transformer structure encoder, a feature difference map processing module, and a lightweight decoder. In the field of CD, this method provides good access to local context information than existing CD methods, other than focusing on global context information. We outperform recent attention-based (STANet and IFNet), Conv Net + transformer-based (BIT), and pure transformer structure (ChangeFormer) methods in terms of F1, IoU score, and overall acquisition. As a result, this study demonstrates that the LeWinTransformer block is well obtained in the hierarchical encoder and feature difference map processing module local context information, which effectively improves CD task performance.

In the future, we will conduct further research on unbalanced sample datasets, inaccurate supervision, and multiple types of changed areas to improve the performance of change detection, as well as improving the ability of the model in real-world scenarios.

## Figures and Tables

**Figure 1:** Overview of the TUNetCD.

**Figure 2:** Feature map partition.

**Figure 3:** FFN.

**Figure 4:** The structure of baseline.

**Table 1:** The average quantitative results of different CD methods on two datasets.

Method		STANet	SNUNet	BIT	ChangeFormer	TUNetCD (ours)
LEVIR-CD	Precision (%)	83.81	89.18	89.24	92.05	**93.23**
	Recall (%)	91.00	87.17	89.37	88.80	**91.98**
	F1 (%)	87.26	88.16	89.31	90.40	**92.36**
	IoU (%)	77.40	78.83	80.68	82.48	**86.22**

DSIFN-CD	Precision (%)	67.71	60.60	68.36	88.48	**88.94**
	Recall (%)	61.68	72.89	70.18	84.94	**85.12**
	F1 (%)	64.56	66.18	69.26	86.67	**87.95**
	IoU (%)	47.66	49.45	52.97	76.48	**76.98**

**Table 2:** Ablation experiment of innovative modules.

Settings		Baseline	Baseline + LeWinTransformer block
LEVIR-CD	Precision (%)	91.65	**93.23**
	Recall (%)	87.50	**91.98**
	F1 (%)	89.53	**92.36**
	IoU (%)	81.04	**86.22**

DSIFN-CD	Precision (%)	87.31	**88.94**
	Recall (%)	82.78	**85.12**
	F1 (%)	84.98	**87.95**
	IoU (%)	73.88	**76.98**

## Data Availability

The data are included within the article.

## Abbreviations

CD: Change detection
BCM: Binary change map
CNNs: Convolutional neural network
FCN: Fully convolutional networks
FC-EF: Fully convolutional early fusion
FC-Siam-Conc: Fully convolutional Siamese-concatenation
FC-Siam-Diff: Fully convolutional Siamese-difference
DSIFN: Deep-supervised image fusion network
NMT: Neural machine translation
NLP: Natural language processing
ViT: Vision transformer
CV: Computer vision
MLP: Multilayer perceptron
DL: Deep learning
STANet: Spatial–temporal attention neural network
ResNet: Residual nets
DASNet: Dual attentive fully convolutional Siamese networks
FP: False positive
FN: False negative
TP: True positive
TN: True negative
P: Precision
R: Recall
IoU: Intersection over Union.
